# Coronavirus pandemic and spirituality in southwest Nigeria: A sociological analysis

**DOI:** 10.1016/j.heliyon.2021.e06451

**Published:** 2021-03-15

**Authors:** Olawale Y. Olonade, Christiana O. Adetunde, Oluwakemi S. Iwelumor, Mercy I. Ozoya, Tayo O. George

**Affiliations:** a Department of Sociology, Covenant University, Ota, Nigeria; b Covenant University Centre for Economic Policy and Development Research (CEPDeR), Nigeria; c Department of Sociology, College of Business and Social Sciences, Landmark University, Nigeria; d School of Social Sciences, Universiti Sains Malaysia, Malaysia

**Keywords:** Coronavirus, Pandemic, Spirituality, Sociology, Analysis, Southwest, Nigeria

## Abstract

**Introduction:**

The coronavirus pandemic outbreak is wreaking much havoc across the globe, with many nations shutting down their economy and social life with the hope of flattening the curve while health practitioners are also gearing efforts in providing a cure for it. Part of the coronavirus challenges is the various spiritual undertones attributed to it in many quarters. Hence, this study seeks to understand the various spiritual undertones attributed to the coronavirus incidence in southwest Nigeria.

**Methodology:**

This paper examined the coronavirus pandemic and spirituality sociologically in southwest Nigeria, using secondary and primary data. Secondary data includes a review of literature, social media comments, official records, and newspaper reports. Primary data entails using google form (questionnaire) circulated via social media with 221 responses retrieved and analyzed using the frequency distribution tables and bar charts. Also, a one-sample t-test was used for further statistical analysis.

**Results:**

Findings show that rather than attributing coronavirus incidence to spirituality alone, most of the respondents also see it as a public health concern, and precautionary measures should adhere. They see the government ban on social gathering, which affected the religious houses as the right thing to do and not solely targeted as religious houses. However, most believe that religious houses provide 'essential' emotional and spiritual support to the people. Respondents also believe they can get their healing from their place of worship even if infected with the coronavirus.

**Conclusion:**

Based on the findings it was recommended that religious organizations should source valid data so that policy-makers can make informed decisions. Also, there is a need to have an accurate record of the number of infected persons and death rates to know the right time to ease lockdown and lift the social gathering measures. There should also be a place for easy and free testing for people. This will help the government ascertain the number of infected persons, reduce the associated fear with the pandemic, and lessen the people's economic, social, and religious effects.

## 1 Introduction

Spirituality and illness are constructs of multidisciplinary interest; hence, beliefs and personal spirituality are primordial concepts found in several health components. According to Roger and Hatala (2017; 6), spirituality is defined as “a dimension of being that gives life meaning through a personal quest for understanding the ultimate questions about life, and about relationships with the sacred or transcendent”. It is also essential to know that spiritual wellbeing is an essential component of individual wellbeing (Chirico, 2016).

Currently, the world is facing a ravaging virus called Coronavirus Disease 2019. It is popularly referred to as (COVID-19). Presently, the pandemic has no cure or actual treatment. The virus has overturned the whole nation, affecting almost all of our habitual social behaviors. Thus, stopping the spread of this infectious disease is paramount in maintaining a healthy society.

While there are substantial numbers of research that have linked religion to health care, others have examined the connection between health and spirituality, its prospect to prevent, cure, or manage ailments (Sloan et al., 1999; Thoresen, 1999; Lukoff et al., 1999; McCullough et al., 2000; Luskin, 2000; Sloan and Bagiella, 2002; Levine and Targ, 2002; Powell et al. 2003).

As posited by Panzini et al. (2007), spirituality serves as a strategy for managing people's life-threatening conditions. It is also a coping mechanism against occupational stress and burnout syndrome in helping professions, including healthcare professionals (Chirico and Magnavita, 2019) and consecrated workers (Chirico, 2017). This is because it gives peace of mind and increases a sense of purpose and meaning of life, often linked to managing anxiety associated with diseases. Personal beliefs define situations of suffering in life. For instance, diseases are referred to as both “spiritual encounters” and physical and emotional experiences. The quest for a purpose in life and the knowledge of connection with God and others appear to be vital to deal with different ailments (Koenig, 2006).

Although several classical studies abound in the literature regarding religion, spirituality, health, and managing with pandemics of transmissible infections like the Plague (Boccaccio, 1886; Defoe, 1722; Mann, 1912), none has explicitly focused on the sociological assessment of COVID-19 regarding spirituality. Recently, Chirico and Nucera (2020) examined the spiritual experience from the coronavirus pandemic but did not cover the disease's social interpretations. Therefore, this study provides a sociological analysis of the relationship between spirituality and COVID-19 in Southwest Nigeria under the following subheadings; COVID-19 and religious/spirituality doctrine, COVID-19 and religious practices, bigoted beliefs associated with COVID-19 and, spiritual struggles. The study further aimed at understanding the various spiritual undertones attributed to the coronavirus incidence in southwest Nigeria.

## 2 COVID-19 and spiritual “Doctrine”

Some Christian doctrines assert that the COVID-19 is apocalyptic and not just ordinary. This belief is widespread in almost all other religious organizations. John of Patmos in 95 AD initiated and wrote this Christian belief. The Book of Revelation accounts for events that will happen at the end of the world. Though no consensus has been reached amongst researchers on interpreting the text, Revelation's book contains these categories; apocalyptic, prophetic, and epistolary.

Especially among the Christian faith, several people have seen Revelation's book as a detailed account of “the end of the world”. In contrast, others perceived it as a manifestation of the heavenly will. The book depicts the four “beasts” that will appear at the end of the world when the seven seals are revealed. Jesus Christ symbolizes the first horseman; battles and killings are represented through the second horseman. In the same vein, the third horseman represents scarcity of food, while the fourth is identified with pandemics and life loss. Some Christians widely believe that the pandemic, as revealed in Revelation's book, precisely, the seven seals signifies the end of the world and that Christ's second coming is about to happen. For this group, COVID-19 has been prophesied in the book of Revelation. The fourth horseman has been related to Coronavirus (Simon et al., 2020).

Some religious groups played significant roles in spreading the virus by neglecting preventive health measures for COVID-19. For example, Rashid (2020) argued that the Shincheonji church in South Korea had contributed majorly to the spread of COVID-19 infections. According to Bostock (2020), this sect is recognized for its aggressive and illusive evangelism. Instructions were given to members to keep their church membership secret while the sect's leader assured the member's direct passage into the “New Earth and the New Heaven”. They shunned preventive care for the virus and were often closely packed during church services. They have also been declining treatment. Roughly 60% of the country's entire infections are said to have emanated from the church (Bostock, 2020).

Another religious organization that neglected the preventive measures are the Haredim in Israel (Halbfinger 2020). This set of people believe in traditional Judaism and firmly hold the Jewish interpretation of the law and customs. They are also against contemporary beliefs and values. They restrict access to people of the world except for commercial activities and essential public relations. Among this group, observing social distancing would be hard, not to talk of other preventive measures because of the country's disturbing poverty level, and many live in congested accommodations. Forward (2020), a Jewish newspaper, reported that although the Haredim make up approximately 12.5% of the nation's population, they constitute about one-third of the country's COVID-19 cases.

More so, as posited by Zevloff (2020), approximately 40% of Bnei Brak residents in Israel may be infected with COVID-19. This could be because they have been encouraged by their spiritual leaders to carry on with life as usual. In March 2020, 400 followers supposedly attended Haredi Rabbi's burial in Bnei Brak (Staff, 2020). Israeli media blamed this group for disobeying government instructions. Their religious beliefs supposedly drive them, saying that they will overcome coronavirus if they study and pray. They see COVID-19 as a reprimand for insufficient religious adherence (Halbfinger, 2020).

Similarly, about 16,000 Muslim hajis in Malaysia were alleged to have spread COVID-19 to six nations while returning home from Tablighi Jamaat, the most prominent Islamic evangelist crusade globally. This crusade emphasized living life during Prophet Muhammad, that is, dining and praying collectively in mosques. Despite the government's clamor against social gatherings, over 8,700 people gathered together to eat and distribute food with one another in bivouacs. One member asserted that: We are only afraid of God and not the fear of coronavirus. A staff of the ministry of health averred that all things be it sound health and illness, are from God. Therefore, anything that occurs to them is known by God (Beech, 2020).

Despite these apocalyptic religious doctrines that have resulted in the spread of the virus, others have offered relief over COVID-19. These include trusting in a loving and caring God, trusting in omniscience, omnipotent God, beliefs in the resurrection of Christ, among others (Simon et al., 2020).

## 3 COVID-19 and religious related practices

Considerably, COVID-19 has affected many religious practices. Important rituals of face-to-face spiritual assemblies have been severely limited; holy pilgrimages were stopped, many schools were closed, group contacts during carnivals and festivities were barred around the globe to prevent the spread of COVID-19.

Religious organizations such as temples, mosques, synagogues, and churches have offered alternative ways of rendering online services through the media such as radio, television, and live streaming. All these alternatives do not provide the benefits of face-to-face communal contact and worship. As such, this does not allow most Christians to partake in the holy communion. According to Simon et al. (2020), car parking lots are used by some Christian organizations for drive-through church services to fill this void. Similarly, mobile apps for prayer and devotionals have been set up by religious leaders/organizations to encourage and keep members close.

Religious practices have changed. Some Roman Catholic bishops suspended the customary obligation of not eating meat during Lent on Fridays throughout the COVID-19 pandemic, which concurred with 2020 Lent (Noori, 2020). Catholic cathedrals demanded that elderly members stay at home and not attend Sunday mass, which usually is obligatory (Parke, 2020). Also, Muslims have been requested to observe prayers at home and postpone Umrah and Haji (Heren, 2020).

As opined by Bentzen (2019), there is a mutual connection between misfortunes and spirituality/religiosity. Once people are faced with calamity, they tend to seek the face of God. One strategy for doing this is through prayer. It is widely accepted that prayer is effective in dealing with adversities. Pargament (1996) stressed that people tend to cope with circumstances beyond their control with God's help.

During this pandemic, it has been proven that there is an increase in prayers and intercessory activities (Coppen, 2020). The United States of American President, Donald Trump, announced March 15, 2020, to seek God in prayer as a national day. There has also been an increase in the search for the term 'prayer' on google. This is said to have continued to increase with every newly recorded case of COVID-19. Likewise, there is a tremendous increase in searching for the keywords Mohammad, Allah, and God. There is speculation that religiosity/spirituality encouraged coping with the plague COVID-19. There is a striking change from congregational prayer to personal prayer with the shutting down of worship places and the lockdown.

A report by Pew Research Center (2020), showed that Americans that had prayed for the COVID-19 to stop would be about 55%. Within this category, 15% are people who 'rarely or by no means ever prayed.' In comparison, those who never practiced any religion that prayed that the virus should stop were estimated to be around 24% (Bentzen, 2019). From the preceding, it is evident that spiritual practices have been altered since the outbreak of coronavirus. Specifically, the face-to-face communal gathering has been stopped; daily online devotion is increasing, while personal commitments also seem to be on the increase (Simon et al., 2020).

## 4 Bigoted beliefs associated with COVID-19

There are widespread monotheistic beliefs that diseases result from sins. Medieval thinkers believed that sicknesses are often trials from God or weapons of punishment. As Pollak (1970) explained, the five means of understanding illnesses are: first, amongst the believer, diseases occur to intensify their faiths by proving their endurance. Second, to protect the righteous against self-esteem. Third, to draw sinners toward repentance. Fourth, for God's glorification due to significant restoration. Fifth, as God's punishment that one has to encounter during one's lifespan.

Recently, fundamentalists, radicalized Catholics, and protestants have publicized their opinions on the internet, saying that COVID-19 is a punishment from God due to numerous sins ranging from homosexuality, wickedness, rape, abortion, paganism to ecological hazard and sorcery. While there are no empirical studies to justify these claims, there is an increase in pastors' accounts on the internet who claimed a connection between transgression and the occurrence of COVID-19 in the past couple of months (Valerio and Heugh, 2020).

For instance, evangelist Franklin Graham asserted that COVID-19 results from the world's disobeying God (Duffy, 2020). Furthermore, Pastor Rick Wiles affirmed that the pandemic has occurred to cleanse the world from iniquities, such as fornication, adultery, and pornographic films on television. Besides, he claims that devoted Christians that believe in Jesus are safe from coronavirus. He enjoined Americans to trace their steps back to God. Pastor Stephen Anderson quoted scriptural verses barring lesbianism, bestiality, and transgender personality (Schlatter, 2010). Pastor Stephen further argued that COVID-19 results from global rebellion against God and states that obeying God will protect the nation against coronavirus.

However, these prevalent opinions of the internet pastors are still vague among Evangelical Christians, with some Christians being warned against relating COVID-19 with sin (Valerio and Heugh, 2020).

Tel Aviv University reported anti-Semitic doctrines, which are now getting more prevalent. Previously, the Jews are accused of causing disasters. For example, one of the anti-Semitic beliefs was that the Jews created the coronavirus to accrue profits from the drug they will produce. They have also been accused of benefitting from the economic meltdown caused by the pandemic. More so, the rejection of Jesu divinity by the Jewish was believed to cause COVID-19. Approximately 18% of anti-Semitic activities have been recorded globally since the outbreak of the COVID-19; this includes; killings, physical assaults on Jews, and demolition of churches and graveyards (Associated Press, 2020).

Another bigotry belief associated with COVID-19 is Christian oppression, which is on the increase in China's current State policy on Atheism. The COVID-19 pandemic is believed to be used by the government to achieve her anti-religious program. One of the churches in Yixing belonging to the Xiangbaishu was destroyed, and a sanctuary in Guiyang Province was defiled by removing the Christian cross from the tower. Also, online streaming, one of the vital means for churches to communicate with their members, was banned in Shandong Region (Parke, 2020). One can draw from the aforementioned that bigotry activities are likely to increase, leading to fear, stress, and psychological trauma (Simon et al., 2020).

## 5 Spiritual struggles

On a final note, it is pertinent to know that this pandemic affects people socially, physically, mentally, spiritually, or religiously. Fear, pressures, anxieties, and disagreements over religious matters are referred to as Spiritual struggles and are not at all unfamiliar with the lifetime (Exline et al., 2014).

Though investigations are still limited on COVID-19, some studies have shown strong relations among distress, natural calamity, and spiritual struggles. Researchers like Pomerleau et al. (2021) have shown that more encounters with significant life events will lead to more significant spiritual struggles, which will, in turn, lead to more significant psychological traumas.

Spiritual struggles come in different ways: One might be angry for been deserted or chastised by God; fears that the illness is as a result of the satanic forces or demonic spirit; doubt the truth about one's spiritual belief; question the purpose and essence of one's life; have difficulties in keeping up with one's ethical standards; and disagreements over spiritual matters (Exline et al., 2014). COVID-19 pandemic has generated quite a lot of these insightful spiritual questions. According to Doehring (2020), COVID-19 incites moral struggles amidst healthcare practitioners who must cope with inadequate medical materials, countless patients, and most uphold their ethical standards not to harm. Perhaps, others might find it hard to sustain their faiths in caring and defending their hope in God with the distress created by the virus.

Furthermore, Pargament and Exline (2021) have linked spiritual struggles to more suffering, physical deterioration, and mental ill-health, as well as the possibility of an increase in the rate of death. Vitorino, Soares, Santo, Lucchetti, Cruz, Cortez, and Lucchetti (2018), also established that spiritual struggles are linked with severe sorrow and exhaustion mal-functioning of the body amongst Brazilian hemodialysis patients. One study recently carried out by Lee (2020) on COVID-19 shows that more spiritual struggles were linked to higher scores on a Coronavirus Anxiety Scale.

## 6 Theory

The Health Belief Model (HBM), developed in the 1950s, is a famous and widely used theory regarding individuals' willingness to procure medical services when experiencing ill-health. The model explains that sick people's decision to seek medical aid depends on the perceived severity of the sickness by the ill person (Rosenstock, 1974). Accordingly, sick people will not seek medical help until they perceive their condition as severe. However, the theory has been criticized for not taking other behavioral factors, such as peer pressure, into consideration (Norman and Conner, 2017).

Nevertheless, the theory has been considered a stable model to explain people's motivation to use medical service during illness. In applying this theory to demonstrate the willingness of sick people in Nigeria to seek medical aid during COVID-19, the idea helps understand that many Nigerians will not use medical services when sick because they are not likely to consider the sickness severe mostly because of their religion. This can be common among Christians, who are told by their leaders that the virus is not real and that even if they are infected by it, God can heal them. As such, their level of spirituality defines their perceived severity of the sickness and, ultimately, their response (see Figure 1).

**Figure 1:** Showing a theoretical framework for HBM.

## 7 Methods

The study adopts a descriptive research design using primary and secondary data collection methods with evidence from scholarly materials and official records. The primary means of data collection include the use of a questionnaire. Two hundred and twenty-one copies of the questionnaire were filled and retrieved from the online Google form. This method was adopted due to the infeasibility of adopting face-to-face administration of copies of a questionnaire in this era of coronavirus pandemic lockdowns. However, the researchers ensure that only respondents who reside in southwest Nigeria filled the questionnaire. The research instrument was a four-point version of the Likert scale style. It contained three main sections that address questions on the fear of COVID-19, Spirituality, and stigmatization. The online google form has been used previously by many researchers on studies of this nature (Lucchetti et al., 2020; Rias et al., 2020; Kowalczyk et al., 2020). The study was conducted in Lagos, Ogun, Oyo, Osun in the southwest part of Nigeria. This area was chosen because of its proximity to Lagos state, regarded as the coronavirus pandemic epicenter (NCDC, 2020). Also, Ogun and Lagos is home to many of the religious bodies' headquarters in Nigeria. Hence, they are likely to be affected by the governments' lockdown measure occasioned by the coronavirus pandemic. The online questionnaire was purposively circulated to adults (18 years and above), who currently reside in Ogun, Lagos, Oyo, and Osun state, through various social media platforms. For data analysis, frequency distribution tables using percentages % and bar charts of the Statistical Package for Social Sciences (SPSS) was used. Also, a one-sample t-test was used for further statistical analysis. Ethical guidelines were duly observed as respondents were informed of the purpose of the study. Also, participation is voluntary, and anonymity is ensured. Ethical approval was obtained from the Covenant University Research and Ethical Committee.

## 8 Results and findings

Table 1 shows the sex distribution of the respondents that were involved in this study. The table shows that 104 (47.1%) of the respondents were male, while the larger 117 (52.9%) were female. This implies that the majority of the respondents surveyed are female. It also shows the marital status distribution of the respondents that were involved in this study. The table shows that Single has 98 (44.35%), Married 116 (52.5%), and Separated/Divorced/Widow 7 (3.2%). By implication, married has the highest number of respondents (see Tables 2 and 3).

**Table 1:** Socio-demographic composition of the respondents.

Question	Responses	Frequency	Percent
Sex	Female	117	52.9
	Male	104	47.1
Marital Status	Single	98	44.3
	Married	116	52.5
	Separated/Divorced/Widow	7	3.2
Religion affiliations	Islam	14	6.3
	Christianity	207	93.7
Age group	18–25	43	19.5
	26–33	96	43.4
	34–41	31	14.0
	41–48	19	8.6
	49–56	14	6.3
	57–65	18	8.1
Education attainment	Secondary Education	25	11.3
	Tertiary Education	196	88.7
	Total	221	100.0
Employment Status	Unemployed	49	22.2
	Self-employed	55	24.9
	Private/Public Sector Worker	117	52.9
Presence of Children	No	116	52.5
	Yes (average = 1)	105	47.5
	Total	221	100.0

Researchers' survey, 2020

**Table 2:** Respondents spiritual perception on COVID-19 pandemic.

Variables	Frequency	Percentage
**I cannot be infected with coronavirus even without adherence to precautionary measures**		
Agree	27	12.2
Disagree	71	32.1
Neutral	17	7.7
Strongly agree	12	5.4
Strongly disagree	94	42.5
**Total**	**221**	**100**

**Coronavirus came as a result of sin**		
Agree	29	13.0
Disagree	42	19.0
Neutral	55	24.9
Strongly agree	8	3.6
Strongly disagree	87	39.4
**Total**	**221**	**100**

**Most victims of coronavirus must have been infected because of their sin**		
Agree	9	4.1
Disagree	55	24.9
Neutral	19	8.6
Strongly agree	8	3.6
Strongly disagree	130	58.8
**Total**	**221**	**100**

**Coronavirus is a punishment from God**		
Agree	30	13.6
Disagree	44	19.9
Neutral	48	21.7
Strongly agree	6	2.7
Strongly disagree	93	42.1
**Total**	**221**	**100**

**Religious houses are the target of government ban on social gatherings**		
Agree	42	19.0
Disagree	59	26.7
Neutral	38	17.2
Strongly agree	9	4.1
Strongly disagree	73	33.0
**Total**	**221**	**100**

**I will rather go to my place of worship for healing rather than isolation centre if confirmed positive of covid19**		
Agree	37	16.7
Disagree	57	25.8
Neutral	32	14.5
Strongly agree	15	6.8
Strongly disagree	80	36.2
**Total**	**221**	**100**

**Religious houses provide 'essential' services to the people**		
Agree	71	32.2
Disagree	47	21.3
Neutral	43	19.5
Strongly agree	29	13.1
Strongly disagree	31	14.0
**Total**	**221**	**100**

Researchers' survey, 2020

**Table 3:** Showing the result of the One-Sample t-test analysis on Coronavirus and Spirituality.

Variables	t	Sig. (2-tailed)	Mean Difference	95% CI
Coronavirus infection without adherence to safety measures	47.730	.000	3.910	3.75–4.07
Coronavirus is related to sin	46.811	.000	3.769	3.61–3.93
Most victims are sinners	76.411	.000	4.394	4.28–4.51
Coronavirus is a punishment from God	48.108	.000	3.846	3.69–4.00
Ban on social gatherings is targeted at religious houses	44.223	.000	3.638	3.48–3.80
Preference for treatment	41.903	.000	3.670	3.50–3.84
‘Essential’ services of religious houses	34.376	.000	2.914	2.75–3.08

The table shows the religious status distribution of the respondents that were involved in the study. Muslims are 14 (6.3%), while Christianity had the highest number of respondents, 93.7% (207). This implies many of the respondents are Christians. It equally shows the distribution of respondents based on age. This shows that 19.5% of the respondents fall within the Age bracket of 18–25years, while 26–33 years constitute 43.4%; 34–41 years 14%; 42–48 years constitute 8.6%; 49–56 years constitute 6.3%, and 57–65 years constitute 8.1%. By implication, the respondents who fall between 26-33 years constitute the larger percentage of the respondents, followed by 18–25years and 34–41 years. It means that many of the respondents are aged and mature enough to have witnessed this era of COVID- 19. According to educational level, those with secondary education fall within the lowest frequency, 23 (11.3%), while those who have gone to tertiary school constitute 88.7%. By implication, respondents' high frequency comes from tertiary education bracket with various qualifications in their chosen field or career.

Still, the table shows that many respondents are working class with 117 frequencies (52.9%) while 22.2% are unemployed. Also, those who engage in self-employment constitute 24.9% (55). By implication, many of the respondents are in the working class and have witnessed several economic and health issues brought about by the pandemic. According to children's presence, the respondents' distribution shows 47.5%, which constitute the largest percentage have children, while 117 (52.5%) are without children (see Figures 2 and 3).

**Figure 2:** Bar Chart showing the relationship between respondents' view on essential nature of religion houses and COVID-19 as a death sentence.

**Figure 3:** Showing the relationship between respondents' treatment preference and government handling of COVID-19 cases.

From the above table supported by the bar charts, 94 of the respondents representing 42.5% and 71 of the respondents representing 32.1% of the respondents, which is the highest strongly disagree and disagree that they cannot be infected with coronavirus even without adherence to COVID-19 precautionary measures while only 27 representing 12.2% and 12 representing 5.4 of the respondents agree and strongly agree that they cannot be infected with coronavirus even without adherence to precautionary measures. Seventeen of the respondents representing 7.7%, however, maintain a neutral stand. This shows that the people of southwest Nigeria believe so much in the coronavirus pandemic's existence and adhere to safety measures to curb its spread.

Whether coronavirus came from sin, 87 of the respondents, representing 39.4%, and 42 of the respondents, representing 19.0%, which are the highest, strongly disagree and disagree respectively that coronavirus results of sin. While 29 of the respondents, representing 13.0%, and 8 of the respondents, representing 3.6%, agree and strongly agree that coronavirus came from sin. Fifty-five of the respondents making 24.9%, were, however, neutral. This finding negates some of the literature reviewed and the position of some religious leaders who have opined that COVID-19 is a result of man's disobedience and a punishment from God (Valerio and Heugh, 2020; Duffy, 2020). However, the result shows that respondents are more informed and understand coronavirus as a public health concern that knows no one and therefore adhered to safety measures.

However, on whether religious houses provide 'essential' services to the people, 71 of the respondents, representing 32.2%, and 29 of the respondents, representing 13.1%, which are the highest agreed and strongly agreed respectively that religious houses provide 'essential' services to the people. While 47 of the respondents, representing 21.3%, and 31 of the respondents, representing 14.0, disagree and strongly disagree that religious houses provide 'essential' services to the people. Forty-three of the respondents, representing 13.1, were, however, neutral. This finding indicates the importance of religious houses by southwest people of Nigeria, known to be either Christian, Muslim or traditional worshippers.

The result above shows that there is a statistical relationship between coronavirus and spirituality, with the P-value of all the variables less than 0.05.

## 9 Discussion

The above findings show that people are adequately aware of the coronavirus pandemic as a public health concern and sin-related. Despite their religious beliefs, they adhere to precautionary measures and do not believe religious houses are the target government ban on social gatherings. However, they believe that religious houses offer ‘essential’ services of providing emotional care and spiritual support to the people and hence, should be opened for worship as many believe they can access healing from their place of worship even if tested positive for coronavirus.

Considerably, COVID-19 has affected many religious practices. Important rituals of face-to-face spiritual assemblies have been severely limited; holy pilgrimages were stopped, many schools were closed, group contacts during carnivals and festivities were barred around the globe to prevent the spread of COVID-19. This, as opined by Exline et al. (2014); (Iwelumor et al., 2020), has resulted in many spiritual struggles of fear, pressures, anxieties, and disagreements over religious matters of which has been predicted will be on the increase by researchers if people are not opportune to worship. Researchers like Pomerleau et al. (2021) have shown that more encounters with significant life events will lead to more significant spiritual struggles, leading to more significant psychological traumas.

Irrespective of this study's findings, the timing of this study posed some limitations as researchers had to rely on the online google form (which is not 100 percent reliable) for data collection because of the lockdown. Therefore, we suggest further research on coping strategies and lived experiences of coronavirus survivals in future research endeavors.

## 10 Conclusions and recommendations

Spirituality is an essential element in the way people face mental health-related problems, such as fear, tensions, anxieties, depression, and post-traumatic stress disorder (PTSD) prevalent with the COVID-19 pandemic. Religious organizations need to source valid data so that policy-makers can make rational decisions. The current lockdown in many places worldwide has caused great hardship for people, both socially, economically, and spiritually. More facts are needed to ascertain how considerable the death rate is, know the number of people who have contacted the virus, see the time to initiate easing of lockdowns, and lift the measure on social distancing. If all these uncertainties could be addressed by putting in place systems that permit easy testing, this might have drastically changed the pandemic's fear and lessened the economic effect, social cost, and religious cost to the people. The media and government also need to maintain accuracy in their reports and curb fake news as much as possible. This will help the people ascertain the pandemic's accurate picture and adhere to appropriate precautionary measures.

## Declarations

### Author contribution statement

Olawale Y Olonade: Conceived and designed the experiments; Analyzed and interpreted the data; Wrote the paper.

Christiana O Adetunde: Conceived and designed the experiments.

Oluwakemi S Iwelumor: Performed the experiments; Wrote the paper.

Tayo O George, Mercy I Ozoya: Contributed reagents, materials, analysis tools or data.

### Funding statement

This research did not receive any specific grant from funding agencies in the public, commercial, or not-for-profit sectors.

### Data availability statement

Data included in supplementary material.

### Declaration of interests statement

The authors declare no conflict of interest.

### Additional information

No additional information is available for this paper.
